The article "Antidiabetic, renal/hepatic/pancreas/cardiac protective and antioxidant potential of methanol/dichloromethane extract of Albizzia Lebbeck Benth. stem bark (ALEx) on streptozotocin induced diabetic rats" was retracted in 2023. Reasons: lack of ethics approval or compliance; concerns about the data; concerns about the images.

# Antidiabetic, renal/hepatic/pancreas/cardiac protective and antioxidant potential of methanol/dichloromethane extract of *Albizzia Lebbeck Benth.* stem bark (ALEx) on streptozotocin induced diabetic rats

**DOI:** 10.1186/1472-6882-14-243

**Published:** 2014-07-16

**Authors:** Danish Ahmed, Vikas Kumar, Amita Verma, Pushpraj S Gupta, Hemant Kumar, Vishal Dhingra, Vatsala Mishra, Manju Sharma

**Affiliations:** 1 Department of Pharmaceutical Sciences, Faculty of Health Sciences, Sam Higginbottom Institute of Agriculture, Technology & Sciences, Deemed University, Allahabad, Uttar Pradesh, India; 2 Department of Pharmacology, Faculty of Pharmacy, Jamia Hamdard, New Delhi, India; 3 Department of Pharmacology, Hamdard Institute of Medical Sciences & Research, Jamia Hamdard, New Delhi, India; 4 Department of Pathology, Moti Lal Nehru Medical College, Allahabad, India

**Keywords:** *Albizzia Lebbeck Benth*, Bark, Diabetes, Streptozotocin, Hypolipidemic, Antioxidant, Histopathology

## Abstract

**Background:**

Hypoglycemic and/or anti-hyperglycemic activities have been recorded with numerous plants, many of which are used as traditional herbal treatments of diabetes. *Albizzia Lebbeck Benth.* stem bark have been used in traditional medicine along with some preliminary reports on its hypoglycemic action. The aim of present investigation was to evaluate the antidiabetic and antioxidant activities of methanolic extract of stem bark of *Albizzia Lebbeck Benth.* in streptozotocin induced diabetic rats.

**Methods:**

The powdered stem bark of *Albizzia Lebbeck Benth.*. was extracted with methanol (MeOH) using soxhlation method and subjected to phytochemical analysis. The methanol/dichloromethane extract of *Albizzia Lebbeck Benth.* (ALEx) was concentrated to dryness using Rotary Evaporator. Diabetes was experimentally induced in the rats by single intraperitoneal administration of Streptozotocin (60 mg/kg). They glycemic control was measured by the blood glucose, glycated heamoglobin and plasma insulin. The oxidative stress was evaluated in the liver and kidney by level of antioxidant markers and various biochemical parameters were assessed in diabetic control and extract treated rats.

**Results:**

Streptozotocin induced diabetic rats depicted the increased blood glucose levels, total cholesterol (TC), triglycerides (TG), low density lipoprotein cholesterol (LDL-c), diminished level of high density lipoprotein cholesterol (HDL-c) level and perturb level of antioxidant markers. Oral administration of MeAL at a concentration of 100, 200, 300 and 400 mg/kg b.w daily for 30 days results a momentous decrease in fasting blood glucose, glycated heamoglobin and enhancement of plasma insulin level as compared with STZ induced diabetic rats. Furthermore, it significantly (p < 0.05) decreased the level of TC, TG, and LDL-c, VLDL-c. While it increases the level of HDL-c to a significant (p < 0.05) level. The treatment also resulted in a marked increase in reduced glutathione, glutathione Peroxidase, catalase and superoxide dismutase and diminished level of lipid peroxidation in liver and kidney of STZ induced diabetic rats. Histopathological studies suggest the diminution in the pancreatic, liver and cardiac muscle damage.

The article "Antidiabetic, renal/hepatic/pancreas/cardiac protective and antioxidant potential of methanol/dichloromethane extract of Albizzia Lebbeck Benth. stem bark (ALEx) on streptozotocin induced diabetic rats" was retracted in 2023. Reasons: lack of ethics approval or compliance; concerns about the data; concerns about the images.

**Conclusion:**

Our research exertion clearly indicates the considerable antihyperglycemic, antihyperlipidemic, antioxidant & pancreas/renal/hepatic/cardiac protective action of ALEx.

## Background

Diabetes mellitus (DM) is the most common endocrine disorder, and affects more than 100 million people worldwide (6% of the population) and in the next 10 years it may affect five times more people than it does now (World Health Organization and American Diabetes Association). The World Health Organization has pointed out that the prevention of diabetes and its complications is not only a major challenge for the future, but essential if health for all is to be an attainable target, and strongly emphasize the optimal, rational use of traditional and natural indigenous medicines (World Health Organization 1985, 1994).

There is an imbalance between radical generating and radical scavenging mechanisms i.e increased free radical production or abridged activity of antioxidant defenses or both results in oxidative stress. Oxidative stress is currently suggested as the mechanism underlying diabetes and diabetic complications [1]. Some of the researches have shown that administration of streptozotocin (STZ) in the animals engender diabetes mellitus and produce an assortment of reactive oxygen species (ROS) as a result of glucose auto-oxidation and protein glycosylation such as superoxide, hydrogen peroxide, and hydroxyl radicals, that are either formed by STZ itself over the short term or result from induced hyperglycemia[2-4]. Additionally, there is a formation of advanced glycation end-products (AGE) by non-enzymatic glycation reactions such as Amadori, Schiff base, and Maillard, persuade the formation of free radical at accelerated rates during the course of diabetes, and are associated with the pathogenesis of chronic diseases such as arthritis, atherosclerosis, and liver cirrhosis [5,6]. Consequently, in recent times, antioxidant therapy has been thought to be effectual for the prevention and treatment of various diseases including diabetes, because oxidative stress plays a key role in the pathogenesis of human diseases [7,8].

The article "Antidiabetic, renal/hepatic/pancreas/cardiac protective and antioxidant potential of methanol/dichloromethane extract of Albizzia Lebbeck Benth. stem bark (ALEx) on streptozotocin induced diabetic rats" was retracted in 2023. Reasons: lack of ethics approval or compliance; concerns about the data; concerns about the images.

*Albizzia Lebbeck Benth.* is a deciduous tree with compound leaves and flat oblong fruits. It is distributed throughout India from the plains upto 900 m in the Himalayas. The bark and flowers of *Albizia Lebbeck Benth*. were used to treat arthritis according to the Siddha system of Medicine [9]. Several studies reported the traditional use of A. Lebbeck Benth. such as the tribal people in Himachal Pradesh and Kashmir use the plant to treat inflammation [10-12], while the tribals of Tamilnadu utilizes the plant in the treatment of bone fractures [13]. Diaorrhea, edema, poisoning, asthma and bronchitis were also being cured by the use of this plant [14,15]. Earlier studies also reported the beneficial effects of A. Lebbeck Benth such as the plant reduces the level of histamine and raised the plasma cortisol in antigen challenged guinea pigs [16] and proves advantageous activity in bronchial asthma patients. [17]. An anti-inflammatory effect of methanolic extract of *Albizia Lebbeck* bark was also reported. [18,19]. The antioxidant potential of leaves of *A. Lebbeck Benth*. was reported by Resmi et al (2006) [20]. Furthermore, a recent research work has reported the hypoglycemic action of *Albizzia Lebbeck Benth.* bark on diabetic rats. The study confirms the improved glycemic control of *Albizzia Lebbeck Benth.* bark [21]. A research work indicating the antidiabetic potential of *Albizzia Lebbeck* bark in alloxan induced diabetic mice was reported [22]. One report portraying the antidiabetic activity of another important species of *Albizzia i.e. Albizzia odoratissima Benth*. in alloxan induced diabetic rats. The study depicted the hypoglycemic potential of Albizzia odoratissima Benth. in diabetic rats [23]*.* The antioxidant action of *Albizzia Lebbeck* leaves on alloxan induced diabetic rats was evidenced by another study, confirming the antioxidant activity of *Albizzia Lebbeck Benth.* on alloxan induced diabetic rats [24]. Some other researches that shows the leaves of plant has the antioxidant potential [25] that can target the free radicals accountable for the destruction of β-cells of pancreas. Consequently, aqueous extract of flowers of *Albizzia Lebbeck* showed enhanced glycemic control in alloxan induced diabetic rats [26].

Despite a long traditional utilization and some reports on the hypoglycemic and antioxidant action of *A. Lebbeck Benth*. in diabetes, no systematic phytochemical and pharmacological research exertion has been carried out on exhaustive research exertion on mode of action, antihyperlipidemic, pancreas, renal, liver and cardiac histopathological alterations, of the methanol/dichloromethane stem bark extract of this impending plant. Therefore, we have taken this research exertion in order to scrutinize plausible mode of action of anti-diabetic potential and the anti-oxidant action and of the *A. Lebbeck Benth.* bark.

The article "Antidiabetic, renal/hepatic/pancreas/cardiac protective and antioxidant potential of methanol/dichloromethane extract of Albizzia Lebbeck Benth. stem bark (ALEx) on streptozotocin induced diabetic rats" was retracted in 2023. Reasons: lack of ethics approval or compliance; concerns about the data; concerns about the images.

## Methods

### Chemicals

Streptozotocin (STZ) was purchased from Sigma Aldrich, St. Louis, USA. The kits for the assay of blood glucose (GLU), total cholesterol(TC), triglyceride(TG), high density Lipoprotein cholesterol(HDL–C), low density lipoprotein cholesterol(LDL–C), hepatic glycogen, hepatic hexokinase, glucose-6-phsophatase, fructose-1-6-bisphosphatase, glucose-6-phosphate, lipid peroxidation (LPO), superoxide dismutase(SOD), catalase (CAT), glutathione Peroxidase (GSH-Px), reduced glutathione (GSH) diagnostic kits were purchased from Span Diagnostics, Surat, India. Glycated serum protein (GSP), blood urea nitrogen (BUN), and creatinine (CRE) diagnostic kits were procured from Accurex, India. Glibenclamide was a generous gift from Ranbaxy Pharmaceutical Company, Gurgaon, India. All other commercial reagents used were of analytical grade.

### Animals

Male albino rats aged between 8-10 weeks (250-300 g) were purchased from Indian Institute of Toxicological Research (IITR), Lucknow, UP, India. Animals were kept in controlled condition in animal house at an ambient temperature of 25-30°C and relative humidity of 55-60% and 12/12 h light/dark cycle and were provided pellet diet along with water *ad libitum*. The experimental protocol has been duly approved by institutional animal ethical committee of Adina Institute of Pharmaceutical Sciences (IAEC Reg. no. 1546/PO/a/11/CPCSEA) and was performed according to the animal ethical guidelines of CPCSEA, government of India.

### Plant material

Fresh stem bark pieces of of A. Lebbeck Benth. were collected from herbal garden of faculty of health sciences, SHIATS, Allahabad, between September 2013-October 2013. The stem barks were identified and authenticated by taxonomist, Botany department in FHS, SHIATS, Allahabad, as stem barks of A. Lebbeck. A voucher specimen of the plant (Ref no. FHS/PHCD/ALB/2013-2014/188) has been deposited in the University’s Botany department herbarium.

### Preparation of plant extracts

The A. Lebbeck Benth. stem barks were chopped into small pieces, powdered, air-dried, sieved (#40) and stored in air tight container at room temperature. Two kilogram of powdered plant material was soaked in 4 L of methanol/dichloromethane in a glass jar for two days at room temperature. The mixture was then subjected to the maceration. The solvent was then filtered with Whatman No. 1. The filtration was repeated 4-5 times until the extract depicts no faint discoloration. The yield of the methanol/dichloromethane extract was found to be 10.82% w/w (132 g). Five grams of this extract were dissolved in 1 mL of dimethyl sulfoxide (DMSO) and then the solution adjusted to 100 mL with distilled water. The extract was further subjected to concentration using a rotary evaporator (Buchi, India) under reduced pressure. The extract was freeze dried for further phytochemical screening.

The article "Antidiabetic, renal/hepatic/pancreas/cardiac protective and antioxidant potential of methanol/dichloromethane extract of Albizzia Lebbeck Benth. stem bark (ALEx) on streptozotocin induced diabetic rats" was retracted in 2023. Reasons: lack of ethics approval or compliance; concerns about the data; concerns about the images.

### Preliminary phytochemicals studies

The extract was subjected to various phytochemicals tests to determine the active constituents present in the crude methanol/dichloromethane leaves extracts of stem bark of A. Lebbeck Benth.

### Acute toxicity study

Acute oral toxicity study was performed according to the 423 guidelines (Acute toxicity class method) lay down by OECD (Organisation of Economic Cooperation and Development). Healthy male albino rats were randomly divided into eight groups with 6 animals in each group. The animals were kept fasting overnight with supplementation of water, thereafter with methanolic/dichloromethane extract of A. Lebbeck Benth. stem bark with increasing doses (100, 200, 300, 400, 500, 600, 700 & 800 mg/kg body weight) with the aid of intragastric tube in order to determine the safe doses by up and down staircase method [27]. The animals were scrutinized continuously for 1 h, then repeatedly for 4 h and later at the end of 24 h for general behavior, autonomic and neurological profiles. Thereafter, one group was administered high dose of A. Lebbeck Benth. extract orally once daily for 20 days and observed for any lethality and death.

### Induction of diabetes

Wistar rats were injected intraperitoneally with STZ dissolved in 0.1 M citrate buffer (pH = 6.5) at 60 mg/kg. Animals of control group were received equal volume of vehicle. After 48 hours of STZ injection, blood glucose of the induced rats was estimated. The rats depicting FBG ≥ 230 mg/dL considered to be diabetic.

### Experimental design

A total of 30 male albino wistar rats were utilized and the animals were randomly divided into 7 groups of 5 animals in each group:

Group I- Normal rats (untreated with dimethylsulfoxide, [DMSO, 3 ml/kg])

Group-II- Diabetic control (administered with Streptozotocin (STZ)

Group-III- Diabetic control + A. Lebbeck Benth. stem bark (ALEx) (100 mg/kg body weight)

Group –IV- Diabetic control + A. Lebbeck Benth. stem bark (ALEx) (200 mg/kg body weight)

Group-V- Diabetic control + A. Lebbeck Benth. stem bark (ALEx) (300 mg/kg body weight)

Group-VI- Diabetic control + A. Lebbeck Benth. stem bark (ALEx) (400 mg/kg body weight)

Group-VII- Diabetic control + Glibenclamide (1 mg/kg body weight)

The extract was administered to the respective groups through oral route using intragastric tube for 45 days.

The article "Antidiabetic, renal/hepatic/pancreas/cardiac protective and antioxidant potential of methanol/dichloromethane extract of Albizzia Lebbeck Benth. stem bark (ALEx) on streptozotocin induced diabetic rats" was retracted in 2023. Reasons: lack of ethics approval or compliance; concerns about the data; concerns about the images.

### Biochemical evaluation

Rats of the different groups were fasted overnight and the blood was withdrawn by retro orbital puncture under light and under anesthesia. Blood was withdrawn from the rats on the 1st, 22nd and 45th day after the induction of diabetes to assess the blood glucose and plasma insulin level by glucose oxidase method [28] and modified method of Herbert et al. (1965) [29] respectively. The alteration in the body weight was observed throughout the therapy in the experimental animals.

At the termination of treatment i.e 45 days, animals were deprived of food for overnight. Activities of hepatic hexokinase, glucose-6-phsophatase, fructose-1-6-bisphosphatase, glucose-6-phosphate were assayed according to the method of Branstrup et al (1957) King (1965), Gancedo and Gancedo (1971) and Robert Langdon (1966), respectively [30-33]. The lipid parameters viz. total cholesterol, HDL cholesterol and triglycerides were evaluated according the method of Zlatkis et al. (1953), Burnstein et al. (1970) and Foster and Dunn (1973), respectively [34-36]. Level of serum LDL cholesterol and VLDL cholesterol were estimated according to the Friedewald formula [37]. Hepatic glycogen level was assessed by the method given by Kemp and Van Hejnigen (1954) [38]. The levels of lipid peroxidation (LPO) in the tissues were evaluated by the method of Okhawa et al. (1979) [39]. Level of superoxide dismutase (SOD) was assayed by the method of Kakkar et al. (1984) [40]. The level of catalase (CAT) enzyme was evaluated by the method of Sinha et al. (1972) [41]. Glutathione Peroxidase (GSH-Px) was assayed by the method given by Rotruck et al. (1973) [42]. Level of reduced glutathione (GSH) was assessed by the method of Ellman (1959) [43].

Levels of blood urea nitrogen (BUN), glycated serum protein (GSP) and creatinine (CRE) in serum were evaluated according to the manufacturer’s instructions provided in diagnostic kits.

### Production of liver and kidney homogenate

For the estimation of the antioxidant level, the rats of the respective groups were kept overnight fasted. All the rats were decapitated and an abdominal incision was performed, in order to harvest liver and pancreas. The whole organs were thoroughly cleaned with chilled normal saline on ice. A 10% (w/v) homogenate of the liver and pancreas (0.03 M sodium phosphate buffer, pH-7.4) was prepared with the help of Ultra-Turrax homogenizer maintaining the speed at 9500 rpm.

### Observation of general condition of rats

The overall general condition of rats such as psychological activity, food intake, water intake, urine output, general locomotor activity, and skin infection were observed every day. The parameters such as body weight and food intake were determined every week.

The article "Antidiabetic, renal/hepatic/pancreas/cardiac protective and antioxidant potential of methanol/dichloromethane extract of Albizzia Lebbeck Benth. stem bark (ALEx) on streptozotocin induced diabetic rats" was retracted in 2023. Reasons: lack of ethics approval or compliance; concerns about the data; concerns about the images.

### Histological assessment of liver, kidney, pancreas and heart sample by heamatoxylin eosin (H/E) staining

At the end of the treatment with the drug, all the rats of different groups were sacrificed using mild anesthesia. After collection of the blood samples, the liver, kidney, pancreas and heart tissues were fixed in neutral formalin solution for 48 hours, dehydrated by passing through graded series of alcohol embedded in paraffin blocks. 4 μm thick sections were prepared using a semi-automated rotator microtome.

### Statistical analysis

Statistical analysis was performed using GRAPH PAD Prism software package, Version 5.0. All the data were expressed as mean ± standard error mean (SEM). The comparisons within groups were evaluated utilizing independent student T-test and one way analysis of variance (ANOVA). The value of p < 0.05 or p < 0.01 were considered to be statistically significant.

## Results

### Effect of ALEx on blood glucose level in normal & STZ induced diabetic treated rats

The biochemical parameters of glycemic control in the animals were summarized in Table 1 (Figure 1). The intraperitoneal administration of streptozotocin (STZ) resulted in nearly 4-fold increase of the fasting blood glucose levels in the male/female diabetic Wistar rats. The blood glucose level was measure at different time intervals during the research exertion viz. on the very first day of induction of diabetes, at the middle of the study i.e. on 21st day and at the finish of the experiment i.e. on 45th day. It was observed that the gradual increase in the dose of the ALEx, the blood glucose level was improvised. At the end of 45 day period, ALEx treated diabetic animals showed a significant reduction of blood glucose nearly to the normal level compared with the diabetic animals (p < 0.05) (Figure 2).

**Table 1:** **Effect of methanol/dichloromethane extract of *Albizzia Lebbeck Benth. *** **stem bark (ALEx) on blood glucose level in normal & STZ induced diabetic treated rats**

**Groups**	**Blood glucose level in mg/dL at different time interval of experimentation**		
	**At start (On 1st day)**	**On 21st day**	**On 45th day**
**Normal rats (untreated with dimethylsulfoxide, [DMSO]) Group 1**	83.78 ± 1.031	86.45 ± 1.003	90.00 ± 0.4292
**Diabetic control (administered with Streptozotocin (STZ) Group 2**	305.4 ± 2.065	317.3 ± 1.612	372.3 ± 2.233
**Diabetic control + (ALEx) (100 mg/kg body weight) Group 3**	295.6 ± 1.842	250.1 ± 2.338^ns^	208.9 ± 0.5738^ns^
**Diabetic control + (ALEx) (200 mg/kg body weight) Group 4**	288 ± 0.4932	235.4 ± 0.8799^ns^	155.7 ± 0.4750
**Diabetic control + (ALEx) (300 mg/kg body weight) Group 5**	283 ± 0.7396	200.2 ± 0.3971*	125.2 ± 1.196*
**Diabetic control + (ALEx) (400 mg/kg body weight) Group 6**	282 ± 0.6635**	166.1 ± 0.7504**	91.68 ± 1.451***
**Diabetic control + Glibenclamide (1 mg/kg b wt.) Group 7**	281.1 ± 0.7859***	157.4 ± 1.004***	86.74 ± 1.701***

The data are expressed as mean ± SEM. (n = number of animals in each group = 5). The comparisons were made by one way ANOVA followed by Dunnent’s test.

ns = non-significant, STZ = Streptozotocin.

*p < 0.05 is considered as significant when compared to the control group (0 h).

**p < 0.001 is considered as very significant when compared to the control group (0 h).

***p < 0.001 is considered as extremely significant when compared to the control group (0 h).

The article "Antidiabetic, renal/hepatic/pancreas/cardiac protective and antioxidant potential of methanol/dichloromethane extract of Albizzia Lebbeck Benth. stem bark (ALEx) on streptozotocin induced diabetic rats" was retracted in 2023. Reasons: lack of ethics approval or compliance; concerns about the data; concerns about the images.

**Figure 1:** **Effect of methanol/dichloromethane extract of *Albizzia Lebbeck Benth. *stem bark (ALEx) on blood glucose level in normal & STZ induced diabetic treated rats.** *p < 0.05 is considered as significant when compared to the control group (0 h); **p < 0.001 is considered as very significant when compared to the control group (0 h); ***p < 0.001 is considered as extremely significant when compared to the control group (0 h).

**Figure 2:** **Effect of Albizia Lebbeck Benth. stem bark extract (ALEx) on histological profile of pancreas in normal, STZ-induced diabetic untreated and STZ-induced diabetic treated wistar rats (Original magnification 10×, DXIT 1200 , Nikon, Japan).** (i) **NPALx**: Heamatoxylin and eosin (H/E) stained sections of pancreas of normal control rat portraying normal islet of langerhans shown by yellow arrows. (ii) **STZP**: Pancreatic section of streptozotocin induced diabetic rat showing no/destroyed islet of langerhans and beta cells depicted by yellow arrows. (iii) **AL100**: Pancreatic section of STZ-induced diabetic rats treated with ALEx at 100 mg/kg body wt. showing small number of islet of langerhans (yellow arrows). (iv) **AL200**: Section of pancreas of STZ-induced diabetic rats treated with ALEx at 200 mg/kg body wt. portraying increased number of islet of langerhans with small proportions of beta cells (yellow arrows). (v) **AL300**: Pancreas of diabetic rats treated with 300 mg/kg body wt. ALEx depicting nearly normal islet of langerhans (yellow arrows). (vi) **AL400**: Sections of pancreas of diabetic treated rats with 400 mg/kg body wt. ALEx showing normal islet of langerhans with numerous beta cells (yellow arrows). (vii) GLP: Pancreatic section of diabetic rats treated with Glibenclamide showing normal pancreatic islet of langerhans with enhancement in the number of beta cells.

The article "Antidiabetic, renal/hepatic/pancreas/cardiac protective and antioxidant potential of methanol/dichloromethane extract of Albizzia Lebbeck Benth. stem bark (ALEx) on streptozotocin induced diabetic rats" was retracted in 2023. Reasons: lack of ethics approval or compliance; concerns about the data; concerns about the images.

### Effect of ALEx on plasma insulin level in normal & STZ induced diabetic treated rats

The level of plasma insulin was measured at different period during the experimentation. A significant decrease in the level of plasma insulin was observed in the diabetic untreated rats compared to the normal rats and the level of plasma insulin was further decreased in the untreated diabetic rats at the end of the study i.e. after 45 days. The treatment with the methanol/dichloromethane extract of ALEx in a dose dependent manner. Treatment with 400 mg/kg body weight of ALEx was shown to produce most significant (p < 0.05) effect on the level of plasma insulin and amplify the level of plasma insulin nearly to the normal as compared to the other doses of ALEx at the end of research exertion (Table 2) (Figure 3).

**Table 2:** **Effect of methanol/dichloromethane extract of *Albizzia Lebbeck Benth. *** **stem bark (ALEx) on plasma insulin level in normal & STZ induced diabetic treated rats**

**Groups**	**Plasma Insulin level in μ at different time interval of experimentation**		
	**At start (On 1st day)**	**On 21st day**	**On 45th day**
**Normal rats (untreated with dimethylsulfoxide, [DMSO]) Group 1**	18.22 ± 0.2077	17.17 ± 0.2059	16.39 ± 0.3864
**Diabetic control (administered with Streptozotocin (STZ) Group 2**	4.31 ± 0.1612	3.27 ± 0.1263^ns^	2.29 ± 0.1619^ns^
**Diabetic control + (ALEx) (100 mg/kg body weight) Group 3**	4.96 ± 0.09011	6.81 ± 0.03929^ns^	6.78 ± 0.1546
**Diabetic control + (ALEx) (200 mg/kg body weight) Group 4**	5.03 ± 0.1771	6.46 ± 0.1928	7.49 ± 0.1608
**Diabetic control + (ALEx) (300 mg/kg body weight) Group 5**	6.68 ± 0.1338	7.59 ± 0.1604	8.29 ± 0.1517*
**Diabetic control + (ALEx) (400 mg/kg body weight) Group 6**	7.79 ± 0.04665*	13.07 ± 0.2095***	15.66 ± 0.1776***
**Diabetic control + Glibenclamide (1 mg/kg b wt.) Group 7**	7.89 ± 0.2871	13.81 ± 0.1706***	16.64 ± 0.1518***

The data are expressed as mean ± SEM. (n = number of animals in each group = 5). The comparisons were made by one way ANOVA followed by Dunnent’s test.

ns = non-significant, STZ = Streptozotocin.

*p < 0.05 is considered as significant when compared to the control group (0 h).

***p < 0.001 is considered as extremely significant when compared to the control group (0 h).

**Figure 3:** **Effect of methanol/dichloromethane extract of *Albizzia Lebbeck Benth. *stem bark (ALEx) on plasma insulin level in normal & STZ induced diabetic treated rats.** *p < 0.05 is considered as significant when compared to the control group (0 h); **p < 0.001 is considered as very significant when compared to the control group (0 h); ***p < 0.001 is considered as extremely significant when compared to the control group (0 h).

The article "Antidiabetic, renal/hepatic/pancreas/cardiac protective and antioxidant potential of methanol/dichloromethane extract of Albizzia Lebbeck Benth. stem bark (ALEx) on streptozotocin induced diabetic rats" was retracted in 2023. Reasons: lack of ethics approval or compliance; concerns about the data; concerns about the images.

### Effect of ALEx on OGTT in normal & STZ induced diabetic treated rats during 120 min (2 h)

The results from the research exertion clearly indicated that the of methanol/dichloromethane extract of *Albizzia Lebbeck Benth.* stem bark (ALEx) (400 mg/kg body weight) and Glibenclamide (1 mg/kg) reduced the blood glucose level (significant hyperglycemia due to administration of glucose load of 2 g/kg p.o) to a significant level (p <0.05) after 2 h of oral administration as compared to the diabetic control (Table 3, Figure 4).

**Table 3:** **Effect of methanol/dichloromethane extract of *Albizzia Lebbeck Benth*. stem bark (ALEx) during 120 min (2 h) on OGTT in normal & STZ induced diabetic treated rats**

**Groups**	**Time (h)**				
	**0 h**	**0.5 h**	**1 h**	**1.5 h**	**2 h**
**Normal rats (untreated with dimethylsulfoxide, [DMSO]) Group 1**	94.03 ± 1.193	135 ± 2.159	144.5 ± 1.385	155.9 ± 1.153	164.8 ± 1.785
**Diabetic control (administered with Streptozotocin (STZ) Group 2**	265.7 ± 1.070	275.9 ± 1.205^ns^	286.4 ± 1.180^ns^	296.6 ± 0.9096^ns^	306.8 ± 0.9778
**Diabetic control + (ALEx) (100 mg/kg body weight) Group 3**	255 ± 1.086	265 ± 0.8882^ns^	273.4 ± 1.024^ns^	283.1 ± 1.020^ns^	292 ± 0.8426^ns^
**Diabetic control + (ALEx) (200 mg/kg body weight) Group 4**	245.2 ± 0.9767	254.8 ± 0.8538	263 ± 1.724**	271.8 ± 1.421	280.4 ± 1.148**
**Diabetic control + (ALEx) (300 mg/kg body weight) Group 5**	234.2 ± 1.263	242.3 ± 1.136**	251.6 ± 0.8199**	261.7 ± 0.9516	270.8 ± 0.6865**
**Diabetic control + (ALEx) (400 mg/kg body weight) Group 6**	217.1 ± 1.329***	240.3 ± 0.4723**	250 ± 0.5276**	258 ± 0.7415	265.3 ± 0.6950***
**Diabetic control + Glibenclamide (1 mg/kg b wt.) Group 7**	221.9 ± 0.6154	242.2 ± 0.6026**	252.1 ± 0.7302***	261.1 ± 0.8815	269 ± 0.5970***

The data are expressed as mean ± SEM. (n = number of animals in each group = 5). The comparisons were made by one way ANOVA followed by Dunnent’s test.

ns = non-significant, STZ = Streptozotocin.

**p < 0.001 is considered as very significant when compared to the control group (0 h).

***p < 0.001 is considered as extremely significant when compared to the control group (0 h).

**Figure 4:** **Effect of methanol/dichloromethane extract of *Albizzia Lebbeck Benth. *stem bark (ALEx) during 120 min (2 h) on OGTT in normal & STZ induced diabetic treated rats.** *p < 0.05 is considered as significant when compared to the control group (0 h); **p < 0.001 is considered as very significant when compared to the control group (0 h); ***p < 0.001 is considered as extremely significant when compared to the control group (0 h).

### Effect of ALEx on weight variation (grams) in normal & STZ induced diabetic treated rats

The body weight variation of the rats was observed at the start and end of the research exertion. As it is obvious from the table (Table 4) (Figure 5), the weight of the diabetic untreated rats was reduced to a significant level. Weight of the ALEx treated rats was increased to a momentous level (p < 0.05) as compared to the normal rats.

The article "Antidiabetic, renal/hepatic/pancreas/cardiac protective and antioxidant potential of methanol/dichloromethane extract of Albizzia Lebbeck Benth. stem bark (ALEx) on streptozotocin induced diabetic rats" was retracted in 2023. Reasons: lack of ethics approval or compliance; concerns about the data; concerns about the images.

**Table 4:** **Effect of methanol/dichloromethane extract of *Albizzia Lebbeck Benth. *** **stem bark (ALEx) on body weight variation (grams) in normal & STZ induced diabetic treated rats**

**Groups**	**Time (h)**	
	**1st Day**	**45th Day**
**Normal rats (untreated with dimethylsulfoxide, [DMSO]) Group 1**	245.6 ± 4.479	297 ± 2.408
**Diabetic control (administered with Streptozotocin (STZ) Group 2**	249.8 ± 3.625	217.2 ± 3.527
**Diabetic control + (ALEx) (100 mg/kg body weight) Group 3**	245.6 ± 1.965^ns^	236 ± 2.702
**Diabetic control + (ALEx) (200 mg/kg body weight) Group 4**	247.4 ± 1.288	247.2 ± 2.417
**Diabetic control + (ALEx) (300 mg/kg body weight) Group 5**	247.2 ± 3.680	266 ± 0.7071
**Diabetic control + (ALEx) (400 mg/kg body weight) Group 6**	252.2 ± 2.245**	300 ± 0.5099**
**Diabetic control + Glibenclamide (1 mg/kg b wt.) Group 7**	249.8 ± 1.020	302 ± 0.7071***

The data are expressed as mean ± SEM. (n = number of animals in each group = 5). The comparisons were made by one way ANOVA followed by Dunnent’s test.

ns = non-significant, STZ = Streptozotocin.

**p < 0.001 is considered as very significant when compared to the control group (0 h).

***p < 0.001 is considered as extremely significant when compared to the control group (0 h).

**Figure 5:** **Effect of methanol/dichloromethane extract of *Albizzia Lebbeck Benth. *stem bark (ALEx) on body weight variation (grams) in normal & STZ induced diabetic treated rats.** *p < 0.05 is considered as significant when compared to the control group (0 h); **p < 0.001 is considered as very significant when compared to the control group (0 h); ***p < 0.001 is considered as extremely significant when compared to the control group (0 h).

### Effect of ALEx on hepatic enzymes in normal & STZ induced diabetic treated rats

Table 5 (Figure 6) portrays the alteration in the activities of carbohydrate metabolizing enzymes in the liver of diabetic control and other experimental animals. The activities of hepatic hexokinase and glucose-6-phosphate dehydrogenase (G6PD) were found to be decreased. On the other hand, the level of gluconeogenic enzymes viz. glucose-6-phosphatase and fructose-6-phosphatase were significantly increased in the diabetic animals compared to those in normal rats. Administration of different doses of ALEx in diabetic rats reversed the alterations in the hepatic enzymes such that animals received 400 mg/kg body weight showed the significant improvement (p < 0.05) in all the hepatic enzymes alterations as compared to the other doses.

The article "Antidiabetic, renal/hepatic/pancreas/cardiac protective and antioxidant potential of methanol/dichloromethane extract of Albizzia Lebbeck Benth. stem bark (ALEx) on streptozotocin induced diabetic rats" was retracted in 2023. Reasons: lack of ethics approval or compliance; concerns about the data; concerns about the images.

**Table 5:** **Effect of methanol/dichloromethane extract of *Albizzia Lebbeck Benth. *** **stem bark (ALEx) on hepatic enzymes in normal & STZ induced diabetic treated rats**

**Groups**	**Biochemical Parameters of Hepatic enzymes**			
	**Hepatic hexokinase (units/min/mg of protein)**	**Gluocse-6-phosphatase (units/min/mg of protein)**	**Fructose 1-6-biphosphatase (units/min/mg of protein)**	**Glucose-6-phosphate dehydrogenase (units/min/mg of protein)**
**Normal rats (untreated with dimethylsulfoxide, [DMSO]) Group 1**	0.214 ± 0.9152	0.176 ± 1.583	0.0282 ± 0.8437	0.128 ± 3.020
**Diabetic control (administered with Streptozotocin (STZ) Group 2**	0.112 ± 1.056	0.273 ± 0.6038	0.0596 ± 1.492	0.058 ± 4.576^ns^
**Diabetic control + (ALEx) (100 mg/kg body weight) Group 3**	0.13 ± 0.9104^ns^	0.241 ± 0.5943^ns^	0.0536 ± 0.6264^ns^	0.0614 ± 3.447
**Diabetic control + (ALEx) (200 mg/kg body weight) Group 4**	0.142 ± 0.2780	0.219 ± 0.3499**	0.0496 ± 0.4148	0.0622 ± 3.083
**Diabetic control + (ALEx) (300 mg/kg body weight) Group 5**	0.17 ± 0.5145	0.197 ± 1.831***	0.0386 ± 0.7895**	0.0892 ± 7.843
**Diabetic control + (ALEx) (400 mg/kg body weight) Group 6**	0.210 ± 0.8454***	0.181 ± 0.8955***	0.0298 ± 1.464	0.122 ± 3.408**
**Diabetic control + Glibenclamide (1 mg/kg b wt.) Group 7**	0.212 ± 0.7552	0.172 ± 0.4005	0.0287 ± 0.8724	0.127 ± 1.711***

The data are expressed as mean ± SEM. (n = number of animals in each group = 5). The comparisons were made by one way ANOVA followed by Dunnent’s test.

ns = non-significant, STZ = Streptozotocin.

**p < 0.001 is considered as very significant when compared to the control group (0 h).

***p < 0.001 is considered as extremely significant when compared to the control group (0 h).

**Figure 6:** **Effect of methanol/dichloromethane extract of *Albizzia Lebbeck Benth. *stem bark (ALEx) on hepatic enzymes in normal & STZ induced diabetic treated rats.** *p < 0.05 is considered as significant when compared to the control group (0 h); **p < 0.001 is considered as very significant when compared to the control group (0 h); ***p < 0.001 is considered as extremely significant when compared to the control group (0 h).

### Effect of ALEx on serum lipid profile in normal & STZ induced diabetic treated rats

As Evident from the Table 6 that diabetic rats exhibited significantly increased serum total cholesterol, VLDL cholesterol, LDL cholesterol, triglycerides and decreased level of HDL cholesterol and hepatic glycogen. Lipid profile of the ALEx treated diabetic rats was significantly improved (p < 0.05) as compared to the untreated diabetic rats (Figure 7).

The article "Antidiabetic, renal/hepatic/pancreas/cardiac protective and antioxidant potential of methanol/dichloromethane extract of Albizzia Lebbeck Benth. stem bark (ALEx) on streptozotocin induced diabetic rats" was retracted in 2023. Reasons: lack of ethics approval or compliance; concerns about the data; concerns about the images.

**Table 6:** **Effect of methanol/dichloromethane extract of *Albizzia Lebbeck Benth.*. stem bark (ALEx) on lipid profile in normal & STZ induced diabetic treated rats**

**Groups**	**Serum lipid profile**				
	**Total cholesterol (TC) (mg/dL)**	**HDL cholesterol (HDL-c) (mg/dL)**	**LDL cholesterol (LDL-c)**	**Triglycerides (TG) (mg/dL)**	**Hepatic glycogen (mg glucose equivalents/mg wet tissue)**
**Normal rats (untreated with dimethylsulfoxide, [DMSO]) Group 1**	128.9 ± 0.3926	53.19 ± 0.4878	27.18 ± 0.5619	77.57 ± 0.5943	49.7 ± 0.2316
**Diabetic control (administered with Streptozotocin (STZ) Group 2**	273 ± 0.7544	14.25 ± 0.2791	105.81 ± 0.8731^ns^	193.1 ± 1.424	17.21 ± 0.09793
**Diabetic control + (ALEx) (100 mg/kg body weight) Group 3**	201.8 ± 0.3189^ns^	15.26 ± 0.1843	82.56 ± 0.4372**	191.7 ± 0.4291	19.17 ± 0.1649
**Diabetic control + (ALEx) (200 mg/kg body weight) Group 4**	188.1 ± 0.4720	28.27 ± 0.5883	81.11 ± 1.201	161.6 ± 0.5797^ns^	25.41 ± 0.4521
**Diabetic control + (ALEx) (300 mg/kg body weight) Group 5**	162.8 ± 0.3100**	34.69 ± 0.5712*	43.94 ± 0.6629	131.3 ± 0.4677	38.41 ± 0.2578*
**Diabetic control + (ALEx) (400 mg/kg body weight) Group 6**	141.4 ± 0.4808***	43.74 ± 0.3495***	30.09 ± 0.3958***	93.57 ± 1.389**	41.68 ± 0.3041***
**Diabetic control + Glibenclamide (1 mg/kg b wt.) Group 7**	145.7 ± 0.5246	48.02 ± 0.1643	28.51 ± 0.7293	81.99 ± 0.5388	48.05 ± 0.1163

The data are expressed as mean ± SEM. (n = number of animals in each group = 5). The comparisons were made by one way ANOVA followed by Dunnent’s test.

ns = non-significant, STZ = Streptozotocin.

*p < 0.05 is considered as significant when compared to the control group (0 h).

**p < 0.001 is considered as very significant when compared to the control group (0 h).

***p < 0.001 is considered as extremely significant when compared to the control group (0 h).

**Figure 7:** **Effect of methanol/dichloromethane extract of *Albizzia Lebbeck Benth. *stem bark (ALEx) on lipid profile in normal & STZ induced diabetic treated rats.** *p < 0.05 is considered as significant when compared to the control group (0 h); **p < 0.001 is considered as very significant when compared to the control group (0 h); ***p < 0.001 is considered as extremely significant when compared to the control group (0 h).

### Effect of ALEx on oxidative stress parameters in normal & STZ induced diabetic treated rats

Table 7 clearly illustrates the effect of ALEx on the antioxidant enzymes. A marked reduction was reported in the level of superoxide dismutase (SOD), catalase (CAT), Glutathione Peroxidase (GSH-Px), and reduced glutathione (GSH) in the STZ induced diabetic rats along with a discernible increase in the level of TBARS. Administration of ALEx at different doses for the 45 days to STZ induced diabetic rats significantly (p < 0.05) increased SOD, CAT, GSH-Px levels with maximum effect seen at 400 mg/kg b.wt. The enhanced level of TBARS was reversed to near normal after administration of ALEx after administering 400 mg/kg b.wt of ALEx. It is pertinent to note that the ALEx was found to be equipped with the antioxidant effect in a dose dependent manner (Figure 8).

The article "Antidiabetic, renal/hepatic/pancreas/cardiac protective and antioxidant potential of methanol/dichloromethane extract of Albizzia Lebbeck Benth. stem bark (ALEx) on streptozotocin induced diabetic rats" was retracted in 2023. Reasons: lack of ethics approval or compliance; concerns about the data; concerns about the images.

**Table 7:** **Effect of methanol/dichloromethane extract of *Albizzia Lebbeck Benth.*. stem bark (ALEx) on oxidative stress parameters in normal & STZ induced diabetic treated rats**

**Groups**	**Oxidative stress**			
	**SOD (units/mg protein)**	**CAT (μ mol/min/mg protein)**	**GSH-px (μ mol/min/mg protein)**	**GSH (mM/100 g tissue)**
**Normal rats (untreated with dimethylsulfoxide, [DMSO]) Group 1**	10.3 ± 0.1642	86.24 ± 0.7028	12.51 ± 0.1523	56.23 ± 0.5273
**Diabetic control (administered with Streptozotocin (STZ) Group 2**	2.67 ± 0.07218	25.28 ± 0.4598	6.274 ± 0.1402	24.58 ± 0.1815
**Diabetic control + (ALEx) (100 mg/kg body weight) Group 3**	3.794 ± 0.1306	26.89 ± 0.3122^ns^	6.628 ± 0.08243	25.7 ± 0.1362
**Diabetic control + (ALEx) (200 mg/kg body weight) Group 4**	6.366 ± 0.01965	38.08 ± 0.4018	7.28 ± 0.01304^ns^	35.69 ± 0.2022
**Diabetic control + (ALEx) (300 mg/kg body weight) Group 5**	7.44 ± 0.1626**	58.61 ± 0.2086**	9.694 ± 0.1273	41.36 ± 0.5254**
**Diabetic control + (ALEx) (400 mg/kg body weight) Group 6**	9.474 ± 0.1209**	75.88 ± 0.6258***	11.64 ± 0.04104***	52.71 ± 0.4298***
**Diabetic control + Glibenclamide (1 mg/kg b wt.) Group 7**	10.41 ± 0.1322	84.3 ± 0.5113	12.53 ± 0.1955	54.52 ± 0.3057

The data are expressed as mean ± SEM. (n = number of animals in each group = 5). The comparisons were made by one way ANOVA followed by Dunnent’s test.

ns = non-significant, STZ = Streptozotocin.

**p < 0.001 is considered as very significant when compared to the control group (0 h).

***p < 0.001 is considered as extremely significant when compared to the control group (0 h).

**Figure 8:** **Effect of methanol/dichloromethane extract of *Albizzia Lebbeck Benth. *stem bark (ALEx) on oxidative stress parameters in normal & STZ induced diabetic treated rats.** *p < 0.05 is considered as significant when compared to the control group (0 h); **p < 0.001 is considered as very significant when compared to the control group (0 h); ***p < 0.001 is considered as extremely significant when compared to the control group (0 h).

### Effect of ALEx on renal function parameters in normal & STZ induced diabetic treated rats

Blood urea nitrogen (BUN), serum creatinine (SCr) and glycated serum protein (GSP), a measurement of kidney function test was evaluated during the experimentation. As it is pertinent from Table 8 that the level of BUN, SCr and GSP increased to a momentous level in the STZ induced diabetic rats. Treatment with different doses of ALEx has profound effect on the altered level of renal function parameters. BUN, SCr and GSP level were decreased to a significant (p < 0.05) level after administration of an assorted doses of ALEx. While the maximum reduction has been observed in the group of rats received 400 mg/kg b.wt. of ALEx as compared to the other doses (Figure 9).

The article "Antidiabetic, renal/hepatic/pancreas/cardiac protective and antioxidant potential of methanol/dichloromethane extract of Albizzia Lebbeck Benth. stem bark (ALEx) on streptozotocin induced diabetic rats" was retracted in 2023. Reasons: lack of ethics approval or compliance; concerns about the data; concerns about the images.

**Table 8:** **Effect of methanol/dichloromethane extract of *Albizzia Lebbeck Benth.*. stem bark (ALEx) on renal function parameters in normal & STZ induced diabetic treated rats**

**Groups**	**Renal function parameters**		
	**Blood urea nitrogen (BUN) (mM/L)**	**Glycated serum protein (GSP) (μ mol/L)**	**Serum creatinine (μ mol/L)**
**Normal rats (untreated with dimethylsulfoxide, [DMSO]) Group 1**	6.54 ± 0.1503	152.3 ± 0.5651	27.35 ± 0.1943
**Diabetic control (administered with Streptozotocin (STZ) Group 2**	13.63 ± 0.1404	313.9 ± 1.426	37.29 ± 0.1431
**Diabetic control + (ALEx) (100 mg/kg body weight) Group 3**	12.11 ± 0.02990^ns^	285.7 ± 1.548^ns^	34.54 ± 0.1297
**Diabetic control + (ALEx) (200 mg/kg body weight) Group 4**	10.53 ± 0.1070	204.1 ± 1.795	33.43 ± 0.1779^ns^
**Diabetic control + (ALEx) (300 mg/kg body weight) Group 5**	8.48 ± 0.1101**	181.9 ± 0.3565*	32.29 ± 0.1512**
**Diabetic control + (ALEx) (400 mg/kg body weight) Group 6**	7.586 ± 0.1244***	162.2 ± 0.6422***	30.24 ± 0.06719***
**Diabetic control + Glibenclamide (1 mg/kg b wt.) Group 7**	7.122 ± 0.03121***	160.8 ± 0.3589***	29.5 ± 0.1336

The data are expressed as mean ± SEM. (n = number of animals in each group = 5). The comparisons were made by one way ANOVA followed by Dunnent’s test.

ns = non-significant, STZ = Streptozotocin.

*p < 0.05 is considered as significant when compared to the control group (0 h).

**p < 0.001 is considered as very significant when compared to the control group (0 h).

***p < 0.001 is considered as extremely significant when compared to the control group (0 h).

**Figure 9:** **Effect of methanol/dichloromethane extract of *Albizzia Lebbeck Benth. *stem bark (ALEx) on renal function parameters in normal & STZ induced diabetic treated rats.** *p < 0.05 is considered as significant when compared to the control group (0 h); **p < 0.001 is considered as very significant when compared to the control group (0 h); ***p < 0.001 is considered as extremely significant when compared to the control group (0 h).

The article "Antidiabetic, renal/hepatic/pancreas/cardiac protective and antioxidant potential of methanol/dichloromethane extract of Albizzia Lebbeck Benth. stem bark (ALEx) on streptozotocin induced diabetic rats" was retracted in 2023. Reasons: lack of ethics approval or compliance; concerns about the data; concerns about the images.

### Effect of ALEx on histopathology of pancreas, kidney, liver and heart

#### Pancreas

Normal control rat exhibited normal histological architecture. Many rounded normal proportions of islet of langerhans were found all around the pancreatic acini. Prominent nuclei with well arranged lobules with surrounding islet cells were found in normal control rats (Figure 2). Groups received STZ, demonstrated cellular damage to the pancreatic acini and islets, which showed pancreatic β-cell damage and degeneration with asymmetrical vacuoles. ALEx treated STZ induced-DM rats showed marked improvement of the cellular injure (Figure 2), as evident from the partial restoration of islet cells, reduced β-cell damage, more symmetrical vacuoles and an increase in number of islet cells.

#### Kidney

Morphological features of kidney remains normal in the control group like prominent glomeruli, collecting ducts, tubules and ascending and descending loops. STZ-induced DM group showed presence of crystal deposition on the glomeruli along with destructed glomeruli and infiltration of red blood cells (Figure 10). Groups received the ALEx demonstrated the reversal of these pathological destructions as apparent by the cell regeneration and removal of crystal deposition.

**Figure 10:** **Effect of Albizia Lebbeck Benth. stem bark extract (ALEx) on histological profile of kidney in normal, STZ-induced diabetic untreated and STZ-induced diabetic treated wistar rats (Original magnification 40×, DXIT 1200 , Nikon, Japan).** (i) **NKALx**: Heamatoxylin and eosin (H/E) stained sections of kidney of normal control rats showing normal glomeruli with normal baseline and tubules (yellow arrows). (ii) **STK**: Section of kidney of STZ-induced diabetic rats depicting destroyed glomeruli with fat deposition on baseline along with infiltration of lymphocytes (yellow arrows). (iii) KAL100: Kidney section of diabetic rats treated with ALEx at dose of 100 mg/kg body wt. portraying improved vasculature and glomeruli (yellow arrows). (iv) KAL200: Section of kidney of diabetic rats treated with 200 mg/kg body wt. of ALEx showing normal tubules along with virtually improved structure of glomeruli. (yellow arrows). (v) KAL300: Kidney section of diabetic treated rats with 300 mg/kg body wt of ALEx depicting nearly normal glomeruli (yellow arrows). (vi) KAL400: Section of kidney of diabetic rat received 400 mg/kg body wt. of ALEx showing normal glomeruli with no infiltration of lymphocytes (yellow arrows). (vii)KGLIB: Section of kidney of the rat supplemented with Glibenclamide showing normal glomeruli with improved structure of tubules (yellow arrows).

The article "Antidiabetic, renal/hepatic/pancreas/cardiac protective and antioxidant potential of methanol/dichloromethane extract of Albizzia Lebbeck Benth. stem bark (ALEx) on streptozotocin induced diabetic rats" was retracted in 2023. Reasons: lack of ethics approval or compliance; concerns about the data; concerns about the images.

#### Liver

The liver cells of normal control groups showed eminent hepatocytes with central vein along with portal triad (Figure 11). The damage to the liver cells in the form of damaged central vein, hepatocytes and portal trial can be clearly seen in the group received STZ. The damage to the liver cells were reversed in the all the ALEx treated groups.

**Figure 11:** **Effect of Albizia Lebbeck Benth. stem bark extract (ALEx) on histological profile of liver in normal, STZ-induced diabetic untreated and STZ-induced diabetic treated wistar rats (Original magnification 40×, DXIT 1200 , Nikon, Japan).** (i) NLALx: Heamatoxylin and eosin (H/E) stained sections of liver of normal control rats showing normal portal triad along with normal hepatocytes with central vein (yellow arrows). (ii) STZL: Liver section of rats received streptozotocin depicting destructed portal trial, disarranged hepatocytes and central vein (yellow arrows).(iii) ALEx100: Section of liver supplemented with 100 mg/kg body wt. of ALEx portaying improvement in structure of portal triad (yellow arrows). (iv)ALEx200: Liver section of rats received 200 mg/kg body wt. of ALEx showing arranged hepatocytes (yellow arrows). (v) ALEx300: Section of liver or diabetic rats treated with 300 mg/kg body wt. of ALEx depicting arranged central vein (yellow arrows). (vi) ALEx400: Liver of diabetic rat showing normal portal traid, central vein and hepatocytes (yellow arrows). (vii) LGLB: Liver section of rat administered with Glibenclamide showing normal microvasculature along with normal hepatocytes (yellow arrows).

#### Heart

Normal control group showed a regular arrangement of cardiac myocytes. STZ-induced DM rats demonstrated a large infarct area with prominent lymphocyte infiltration and fibrosis. Administration of ALEx reversed these morphological changes in dose dependent manner (Figure 12).

**Figure 12:** **Effect of Albizia Lebbeck Benth. stem bark extract (ALEx) on histological profile of heart in normal, STZ-induced diabetic untreated and STZ-induced diabetic treated wistar rats (Original magnification 40×, DXIT 1200 , Nikon, Japan).** (i) NHALx: Heamatoxylin and eosin (H/E) stained sections of heart (oblique cut) of normal control rats showing well arranged cardiac myocytes and normal striations (yellow arrows). (ii) STZH: Section of heart of STZ-induced diabetic rats depicting disarranged cardiac myocytes with destroyed striations (yellow arrows). (iii) ALEx100: Cardiac section of rats received 100 mg/kg body wt. of ALEx portraying better striations (yellow arrows). (iv) ALEx200: Heart section of diabetic rats administered with 200 mg/kg body wt. of ALEx showing improved arrangement of cardiac myocytes (yellow arrows). (v) ALEx 300: Section of heart of diabetic rats supplemented with 300 mg/kg body wt. of ALEx, showing nearly normal cardiac myocytes and striations (yellow arrows). (vi) ALEx400: H/E stained section of heart of diabetic rats received 400 mg/kg body wt. of ALEx depicting normal arrangement of cardiac myocytes and normal striations (yellow arrows). HGLB: Heart section of diabetic rats administered with Glibenclamide portraying normal cardiac myocytes (yellow arrows).

The article "Antidiabetic, renal/hepatic/pancreas/cardiac protective and antioxidant potential of methanol/dichloromethane extract of Albizzia Lebbeck Benth. stem bark (ALEx) on streptozotocin induced diabetic rats" was retracted in 2023. Reasons: lack of ethics approval or compliance; concerns about the data; concerns about the images.

## Discussion

The present research exertion was designed to evaluate the prospective effects of *Albizzia Lebbeck Benth.* stem bark extract (ALEx) on glycemic control, antioxidant status and its histopathological changes on the liver, pancreas, kidney and heart. STZ diabetic model is one of the important and most widely accepted and utilized method to induced diabetes comparable to human diabetes. At present, a growing apprehension has attracted attention of many researchers to and has brought back traditional and complementary medicine due to their pharmacological and economic advantages [44-46]. Our previous research work also depicts the protective effect of one traditionally used polyherbal formulation against the diabetes induced liver and pancreatic damage [47].

Streptozotocin enters the pancreatic β-cells through one of the important glucose transporter known as GLUT 2 and damages the β-cells by DNA alkylation. Furthermore, the damage is also done by the production of superoxide radicals inside the β-cells which are produced with the help of xanthine oxidase. In addition to the following mechanism another important mechanism by which the β-cells are partially destroyed are the formation of nitric oxide free radicals. Therefore, free radicals play an important role in the development of diabetes mellitus by causing the partial destruction of β-cells [48]. In view of that, we hypothesized that free radicals scavenging properties of a compound can ameliorate the diabetic conditions.

Flavonoids are naturally occurring phenolic compounds that are found in plants. They are widely distributed in most of the frequently consumed beverages and food products of plant origin such as fruits, vegetables, tea, wine and cocoa [49]. In recent years much of the attraction was on the antioxidant activity of flavonoids, due to their ability to reduce the free radicals formation and to scavenge free radicals. There are strong experimental evidences that show that patients with diabetes mellitus are susceptible to increase in blood level of oxidants [50,51].

An enhancement of blood glucose level was observed in the oral glucose tolerance test (OGTT) was considerably greater in the STZ induced diabetic rats as compared to the non-diabetic rats. The level of plasma insulin was increased in the non-diabetic rats as compared to the diabetic rats in which there is a decrease in the plasma insulin level. Administration of ALEx at different dose noticeably enhanced the impaired glucose tolerance in the STZ induced diabetic rats with improvement in the plasma insulin level. Based on the above results, the hypoglycemic action of the *Albizzia Lebbeck Benth.*. stem bark extract may be due to the insulin like action i.e performing its action at the peripheral level to improve the cellular uptake of glucose or enhance the glycogenesis. Many of the plant and their extracts have shown to exert hypoglycemic action through stimulation of insulin release [52,53]. The hypoglycemic action of the ALEx is comparable to the conventional sulfonylurea i.e. Glibenclamide that is reported to enhance the insulin release from the beta cells of pancreas though their activation. Therefore, it is presupposed that ALEx could be accountable for potentiation of the pancreatic secretion of insulin from regenerated β-cells by inhibiting ATP sensitive K + channels like Glibenclamide for stimulation of insulin from the pancreatic beta cells.

The article "Antidiabetic, renal/hepatic/pancreas/cardiac protective and antioxidant potential of methanol/dichloromethane extract of Albizzia Lebbeck Benth. stem bark (ALEx) on streptozotocin induced diabetic rats" was retracted in 2023. Reasons: lack of ethics approval or compliance; concerns about the data; concerns about the images.

Diabetic state is characterized by a severe loss in body weight because of loss or degradation of structural proteins [54]. Due to insulin deficiency there is a marked reduction in the protein content in the muscular tissue due to proteolysis [55]. The reversal in loss of weight in the ALEx treated diabetic rats group exhibited that restoration of the weight loss may be due the reversal of proteolysis, gluconeogenesis and glycogenolysis [56].

In experimental diabetes, there is a marked alteration of the enzymes accountable for glucose metabolism. Persistent hyperglycemia is the major factor responsible for such metabolic alterations that lead to the development of diabetic complications such as neuropathy and micro-vascular complications [57]. Hepatic Hexokinase and glucose-6-phosphate dehydrogenase activities have been found to be decreased in the diabetic rats, which may be due to the insufficiency of insulin. Hexokinase is one of the important enzyme responsible for phosphorylation of glucose into glucose-6-phosphate [58].

Insufficiency of hexokinase results in decreased glycolysis and a marked reduction in the utilization of glucose for the production of energy. Oral administration of ALEx to diabetic rats resulted in considerable increase in the activity of hexokinase in dose dependent manner (Table 5).

The activities of hepatic glucose-6-phosphatase as well as fructose-1,6 biphosphatase were increased to a significant extent in STZ induced diabetic rats. The above mentioned enzymes are the key regulators in gluconeogenic pathway. The increased activities of the two enzymes may be due to the increased synthesis of enzymes contributing to the enhanced glucose production by the liver in the period of diabetes [59]. In our research exertion, administration of ALEx had a significant effect on the level of glucose-6-phosphatase and fructose-1,6 biphosphatase, which decreased to considerable level in dose dependent manner. Maximum effect was observed in 400 mg/kg body weight. The reduction in the above two biochemical enzymes portrays the sequential metabolic correlation between increased glycolysis and decreased glyconeogenesis.

The article "Antidiabetic, renal/hepatic/pancreas/cardiac protective and antioxidant potential of methanol/dichloromethane extract of Albizzia Lebbeck Benth. stem bark (ALEx) on streptozotocin induced diabetic rats" was retracted in 2023. Reasons: lack of ethics approval or compliance; concerns about the data; concerns about the images.

In the pathogenesis of diabetes, lipid plays a significant factor. Increased level of cholesterol and lipids in plasma represent a risk factor for coronary artery disease [60].

Increased level of total cholesterol, triglycerides, low density lipoprotein cholesterol (LDL-cholesterol), very low density lipoprotein cholesterol (VLDL-cholesterol) was observed in streptozotocin induced diabetic rats. Hypercholesterolemia in the rats received streptozotocin is caused by increased intestinal absorption and increased cholesterol biosynthesis [54]. Treatment with ALEx reduced the total cholesterol, LDL-c, VLDL-c and triglycerides level to a significant extent in dose dependent manner, while increasing the beneficial HDL level to a considerable extent. It is assumed that ALEx may exert its hypocholesterolemic effect either due to decreased intestinal absorption or decreased cholesterol biosynthesis. The lipoproteins in the diabetic rats are oxidized and may be cytotoxic, which can be reversed by the administration of antioxidants [61]. Our results clearly demonstrated that ALEx recovered the imbalanced lipid profile of STZ induced diabetic rats in dose dependent manner.

Antioxidant capacity is reduced to a significant extent in the plasma of STZ-induced diabetic rats, due to the higher requirement of antioxidants in order to regulate the reactive oxygen species (ROS) homeostasis [62]*.* Nevertheless, enhanced plasma antioxidant capacity in conjunction with reduced lipid peroxidation could be attained by regular ingestion of rich source of antioxidant compounds. In our research exertion, we examined the antioxidant capacity of ALEx. ROS can be primarily eliminated by essential free radical scavenger enzymes, such as superoxide dismutase (SOD), catalase (CAT), glutathione (GSH) and glutathione Peroxidase (GSH-Px). As it is obvious from the Table 7 that activities of antioxidant related enzymes were detiorated by administration of streptozotocin (STZ). When the activities of these important antioxidant enzymes were diminished, the superoxide anion and hydrogen peroxide (H_2_O_2_) radical are available in excess, prompting the production of ROS and dissemination of lipid peroxidation. The level of SOD, CAT, GSH, GSH-Px were diminished in all the tissue of diabetic individuals [63]. Supplementation of ALEx in STZ induced diabetic rats protect, to certain degree, further improvement in the activities of GSH, GSH-Px, CAT and SOD in liver of the diabetic rats.

The article "Antidiabetic, renal/hepatic/pancreas/cardiac protective and antioxidant potential of methanol/dichloromethane extract of Albizzia Lebbeck Benth. stem bark (ALEx) on streptozotocin induced diabetic rats" was retracted in 2023. Reasons: lack of ethics approval or compliance; concerns about the data; concerns about the images.

Diabetic nephropathy (DN) is one of the major micro-vascular complications of diabetes mellitus. In our present research study, the development of DN is confirmed by significant enhancement in the level of blood urea nitrogen (BUN), glycated serum protein (GSP) and serum creatinine (Scr). Supplementation of ALEx in dose dependent manner improves the renal function parameters. Effect of ALEx 400 mg/kg body weight on reducing oxidative stress and renal function parameters was significantly (p < 0.05) better than the other doses.

Histopathological examination of diabetic pancreas, showed islet of langerhans with fatty infiltration and damaged acini. Administration of ALEx restores the morphological changes in the pancreas to normal. Similarly, the microscopic sections of STZ-diabetic liver demonstrated the damaged central vein and surrounding portal triad. Supplementation of ALEx at different dose recovers the normal histology of liver. Furthermore, the damaged glomeruli, tubules, collecting ducts and ascending and descending limbs were seen the kidney of STZ-induced diabetic rats. These destructive morphological changes were upturned to normal in all ALEx treated groups. Correspondingly, arranged cardiac myocytes were observed in the ALEx supplemented groups as compared to the toxic diabetic rats. According to the microscopic examinations, the severe hepatic, renal, pancreatic and cardiac lesions induced by STZ were significantly diminished and restored by administration of ALEx at lower to higher doses.

## Conclusion

The results of the present investigation indicate that ALEx ameliorates the hypoglycemia mediated oxidative stress as well as corrects the lipid profile, hepatic and renal parameters, which was evidenced by improved glycemic control, lipid, renal, hepatic as well as antioxidant biochemical parameters. It can also be concluded that ALEx is a good source of natural antioxidants, which could be a valuable tool in controlling lipid peroxidation and maintaining lipid and lipoproteins. The histological and ultra-structural observations made on the pancreas, liver, kidney and heart tissue substantiate that ALEx protects the oxidative damage of islets of langerhans, hepatocytes, glomeruli and cardiac myocytes on account of its antioxidant potential. Consequently, further studies on the isolation of active principle (s) which exerts the anti-diabetic, hepatic and renal protective effect from ALEx are at the developmental stage in our laboratory.

The article "Antidiabetic, renal/hepatic/pancreas/cardiac protective and antioxidant potential of methanol/dichloromethane extract of Albizzia Lebbeck Benth. stem bark (ALEx) on streptozotocin induced diabetic rats" was retracted in 2023. Reasons: lack of ethics approval or compliance; concerns about the data; concerns about the images.

## Competing interests

The authors declare that they have no competing interests.

## Authors’ contributions

DA and MS carried out the experimental work, biochemical and statistical analysis. VK, AV & PSG designed and planned the study as well as drafting and revision of the manuscript. HK, VD & VM performed the histological study, interpretation and analysis work. All authors read and approved the manuscript.

## Pre-publication history

The pre-publication history for this paper can be accessed here:

http://www.biomedcentral.com/1472-6882/14/243/prepub
